The article "Overexpression of Cosmc suppresses cell migration and invasion in different subtypes of breast cancer cells via Tn and T glycans" was retracted in 2022. Reasons: contaminated cell lines or tissues; duplicated images; signs of a paper mill; unreliable results or conclusions.

# Overexpression of Cosmc suppresses cell migration and invasion in different subtypes of breast cancer cells via Tn and T glycans

**DOI:** 10.1042/BSR20191062

**Published:** 2020-06-17

**Authors:** Jun Liu, Feng Xu, Jie Li, Hongchuan Jiang

**Affiliations:** Department of Breast Surgery, Beijing Chao-Yang Hospital, Capital Medical University, Beijing 100043, P.R. China

**Keywords:** Apoptosis, Breast cancer, Cosmc, Metastasis, Proliferation, Tn and T glycans

## Abstract

**Objectives:** The high mortality of breast cancer (BC) is associated with the strong metastatic properties of primary breast tumor cells. The present study was conducted in order to clarify the effect of Cosmc on the growth and metastasis of BC cell lines of different molecular types, which may be implicated in the regulation of Tn and T glycans.

**Methods:** BC cell lines with different molecular types were transduced with shRNA targeting Cosmc or, Cosmc overexpression plasmid in order to explore the role of Cosmc in cell proliferation, migration, invasion, and apoptosis. The protein levels of Tn, T, Cosmc, proliferation-related factors (Ki67 and PCNA) and apoptosis-related factors (Bax and Bad) in BC cell lines were determined by Western blot analyses. Finally, the role of Cosmc was substantiated through *in vivo* experiments.

**Results:** Cosmc was down-regulated in different subtypes of BC cell lines compared with normal control cells. Overexpression of Cosmc suppressed the proliferation, migration, and invasion, yet promoted the apoptosis of BC cells, as reflected by *in vitro* experiments. Additionally, *in vivo* tumor xenografts in nude mice showed that ectopic overexpression of Cosmc inhibited the tumor growth of BC cells. Consequently, the levels of proliferation-related factors and Tn antigen were decreased, while those of apoptosis-related factors and T antigen were increased in BC cells. This observation was confirmed *in vivo* in xenograft tumors.

**Conclusion:** Collectively, up-regulation of Cosmc potentially impedes BC growth and metastasis by modulating the balance between Tn and T glycans.

## Introduction

Breast cancer (BC) is the most frequently occurring cancer among women and its incidence worldwide is on the rise [1], due to insufficiencies in early detection, as well as many patients that do reach a metastatic stage end up succumbing to death [2]. According to a 2015 estimate, 270,000 women were newly diagnosed with BC in China, ultimately leading to 70,000 deaths within the same year [3]. Mastectomy in combination with radiotherapy remains the most effective therapeutic options for the majority of patients with BC, resulting in a relatively promising outcome [4]. However, the lack of in-time interventions for invasive and metastatic behaviors of BC cells eventually results in invasion and metastasis, which is the final and fatal stage of BC progression [5]. Hence, a better understanding of the mechanisms governing the signaling pathways orchestrating tumor angiogenesis in BC should been thoroughly explored.

The article "Overexpression of Cosmc suppresses cell migration and invasion in different subtypes of breast cancer cells via Tn and T glycans" was retracted in 2022. Reasons: contaminated cell lines or tissues; duplicated images; signs of a paper mill; unreliable results or conclusions.

Cosmc, as an endoplasmic reticulum chaperone required for the expression of T antigen, is essential for normal protein O-GalNAc glycosylation; meanwhile its loss-of-function could lead to the Thomsen nouvelle (Tn) antigen expression [6]. O-glycans include Tn antigen, sialyl-Tn (sTn), and the Thomsen-Friedenreich (TF or T) antigen; however, aberrant O-glycosylation is often observed on the tumor cell surface and is related to poor prognosis in patients with cancer [7]. The presence of abnormal O-glycans, such as enrichment of Tn antigen, has been found in over 90% of breast cancers. Furthermore, breast cancer progression is delayed after removal of the core 1-derived O-glycans and subsequent expression of Tn in mammary epithelial cells as seen in the spontaneous BC mouse model [8]. Prior evidence has indicated that silencing of Cosmc was found to modulate abnormal O-glycosylation, which contributed to oncogenic activities in pancreatic cancer [9]. Moreover, impaired Cosmc has been identified in colorectal cancer tissues according to bio-functional investigations conducted in a previous study [10]. Therefore, we hypothesized that Cosmc may participate in the development of BC by modulating the balance between Tn and T glycans. In the present study, we aim to investigate the effects of Cosmc on the growth and metastasis of BC cells via regulation of Tn and T glycans.

## Materials and methods

### Western blot analysis

Total protein from BC and adjacent normal tissues or from cell lines, were extracted, separated by polyacrylamide gel electrophoresis (PAGE) and transferred onto a polyvinylidene fluoride (PVDF) membrane through the wet transfer method. Next, the membrane was blocked in 5% bovine serum albumin (BSA) for 1 h and then probed with primary rabbit anti-human antibodies against Cosmc (sc-271829, Santa Cruz, California, U.S.A.), Ki67 (ab92742, 1:5000), proliferating cell nuclear antigen (PCNA; ab152112, 1:1500), Bcl-2-associated X protein (Bax; ab32503, 1:5000), and Bad (ab32445, 1:3000) (Cambridge, MA, U.S.A.) at 4°C overnight. The next day, the membrane was washed with Tris-Buffered Saline Tween-20 (TBST) (5 min× 3 times), and incubated with horseradish peroxidase-labeled goat anti-rabbit IgG (ab205718, 1:20,000) for 1 h. After development, ImageJ 1.48u software (National Institutes of Health, Bethesda, MA, U.S.A.) was used for protein quantitative analysis.

The article "Overexpression of Cosmc suppresses cell migration and invasion in different subtypes of breast cancer cells via Tn and T glycans" was retracted in 2022. Reasons: contaminated cell lines or tissues; duplicated images; signs of a paper mill; unreliable results or conclusions.

### Cell culture and lentiviral vector construction

The normal human mammary epithelial cell line (HMEC) HBL-100 and four BC cell lines with different molecular types (luminal A: MCF-7, luminal B: BT474, HER-2 enriched: MDA-MB-453, Triple-negative: MDA-MB-231) from American Type Culture Collection (Manassas, VA, U.S.A.) were cultured with medium containing 15% fetal bovine serum (FBS), and incubated in 5% CO_2_ at 37°C. The full-length complementary DNA (cDNA) sequence of Cosmc (from the Ensemble database) and its negative nonsense control sequences were designed by Ambion’s lentiviral vector Designer. The construction and sequencing identification of lentiviral interference vector and shRNA vector were entrusted to Shanghai Genechem Co., Ltd. (Shanghai, China).

### Cell treatment

The BC cell lines in the logarithmic growth phase were plated into a 24-well plate. When the cell confluence reached 50%, 1 μl lentiviral solution of oe-Cosmc, sh-Cosmc, oe-Cosmc NC and sh-Cosmc NC was added for 24 h. Then, the medium was changed and the cells were further cultured at 5% CO_2_ at 37°C for 48 h. BC cell lines with stable overexpression or, low expression of Cosmc, were selected. BC cell lines (MCF-7 and BT474) with a high expression of Cosmc were grouped into sh-NC (cells transduced with sh-Cosmc NC lentiviral vector) and sh-Cosmc (cells transduced with sh-Cosmc lentiviral vector) groups; and those with a poor expression of Cosmc (MDA-MB-453, MDA-MB-231) were assigned into overexpression (oe)-NC (cells transduced with oe-Cosmc NC lentiviral vector) and oe-Cosmc (cells transduced with oe-Cosmc lentiviral vector) groups.

### 5-ethynyl-2′-deoxyuridine (EdU) staining

The cells were incubated in the culture medium containing EdU solution (C10341-1, RiboBio Co., Ltd., Guangzhou, Guangdong, China) for 2 h, and then fixed with PBS containing 4% paraformaldehyde for 15 min at room temperature. Next, PBS containing 0.5% Triton-100 was added to the cells for 20-min incubation at room temperature. Afterward, the cells in each well were treated with 100 µl staining solution for 30 min at room temperature avoiding exposure to light followed by nuclear staining with 4′,6-diamidino-2-phenylindole (DAPI) for 5 min. Finally, the cells were observed and photographed under a fluorescence microscope (FM-600, Shanghai Pudan Optical Instruments Co., Ltd., Shanghai, China). The cells were photographed from the perspective of 6–10 randomly selected view fields to count the number of positive cells in each field: the rate of EdU labeling (%) = positive cell number / (number of positive cells + number of negative cells) × 100%.

The article "Overexpression of Cosmc suppresses cell migration and invasion in different subtypes of breast cancer cells via Tn and T glycans" was retracted in 2022. Reasons: contaminated cell lines or tissues; duplicated images; signs of a paper mill; unreliable results or conclusions.

### Scratch test

The cells transduced with lentiviral vectors were incubated in a 5% CO_2_ incubator at 37°C for 24 h, and a horizontal scratch was made on the single layer of cells with a 10 μl pipette tip. The cells were then incubated with serum-free medium for 24 h. Cell migration was observed at the 0th and 24th h under an inverted microscope. Three views were selected in each group for photographs and the relative distance between the cells on both sides of the scratch was measured using the formula: relative migration distance of the cells = the distance difference/2. The cell relative migration rate = relative migration distance/the distance from the scratch edge to the scratch midline at the 0th h.

### Transwell assay

The cells were diluted with 100 μl serum-free medium to prepare cell suspension (1 × 10^6^ cell/ml), which was inoculated into the apical chamber of Transwell chamber (3413, Beijing Unique Biotechnology Co., Ltd., Beijing, China) coated with Matrigel (40111ES08, Yeasen Biotechnology Co., Ltd., Shanghai, China) diluted by serum-free DMEM at a ratio of 1:2, and incubated at 37°C for 4–5 h. Next, 500 μl DMEM containing 20% FBS was added to the basolateral chamber. Triplicate wells were set for each group. The cells were incubated in 5% CO_2_ at 37°C for 24 h. The Transwell chamber was fixed with 5% glutaraldehyde at 4°C, and stained with 0.1% Crystal Violet for 5 min. Cotton balls were used to wipe off the cells on the inner surface of the chamber. Finally, the cells were observed under an inverted fluorescence microscope (TE2000, Nikon Corporation, Tokyo, Japan). Five visual fields were photographed randomly, and the average number of cells invaded through the chamber was quantified in each group.

### Flow cytometry

The cells were treated with ethylenediaminetetraacetic acid (EDTA)-free trypsin, and centrifuged, after which cell apoptosis was detected according to the instructions of a Annexin-V-fluorescein isothiocyanate (FITC) cell apoptosis detection kit (Sigma-Aldrich Chemical Company, St Louis, MO, U.S.A.). In brief, the Annexin-V-FITC, propidium iodide (PI), and 4-(2-hydroxyethyl)-1-piperazineëthanesulfonic acid (HEPES) solution were formulated into Annexin-V-FITC/PI dye solution at a ratio of 1:2:50. A total of 1 × 10^6^ cells was resuspended with 100 μl dye solution and incubate for 15 min at room temperature. Then, the cells were treated with 1 ml HEPES solution, and mixed. Finally, the bandpass filters of 525 and 620 nm were activated by 488 nm wavelength of light to detect FITC and PI fluorescence for cell apoptosis. The rate of cell apoptosis was calculated by FITC minus PI.

Tn and T activity detection: The cultured cells (1 × 10^5^) were resuspended in 100 µl PBS containing 0.5% BSA at 37°C for 30 min, and then incubated with VVA lectin-FITC and PNA lectin-FITC (Vector Laboratories) at 1:100 in PBS with 0.5% BSA on ice for 30 min. After washing twice, the fluorescence intensity of 1 × 10^4^ cells per sample in 100 μl PBS was analyzed by flow cytometry (FACS Calibur, BD Pharmingen).

The article "Overexpression of Cosmc suppresses cell migration and invasion in different subtypes of breast cancer cells via Tn and T glycans" was retracted in 2022. Reasons: contaminated cell lines or tissues; duplicated images; signs of a paper mill; unreliable results or conclusions.

### Tumor xenografts in nude mice

In total, 48 BALB/c nude mice (aged 4–6 weeks and weighing 16–20 g; Shanghai Lingchang Biological Technology Co., Ltd., Shanghai, China) were fed at specific pathogen-free (SPF) grade environment of Animal Experimental Center of Xiangya Medical College (No. 159). BALB/c nude mice were fed with sterile food and water, with a 12-h light/dark cycle for adaptive 7 days. The mice (6 from each group) were subsequently injected with BC cells transduced with lentiviral vectors, and then tumor growth was observed and recorded on the 7th, 14th, 21st and 28th day. The short diameter (*a*) and long diameter (*b*) of the tumor were recorded, and the tumor volume = π(2*ab*)/6. Moreover, all the detections were carried out under light. Each measurement was repeated three times. On the 28th day, the nude mice were euthanized by carbon dioxide asphyxiation after being anesthetized with pentobarbital sodium (40 mg/kg) [11] and tumors were collected.

### Statistical analysis

Statistical analysis was performed using SPSS 21.0 statistical software (IBM, Armonk, N.Y., U.S.A.). Measurement data were presented as mean ± standard deviation. Differences between two groups were analyzed using non-paired *t*-test. One-way analysis of variance (ANOVA) with Tukey’s post hoc test was used for comparisons among multiple groups. Repeated measures ANOVA with Bonferroni post hoc test was used for comparisons at different time points. A *P* value < 0.05 indicated statistical significance.

## Results

### Cosmc is poorly expressed in BC cell lines

Four BC cell lines with different molecular types (Luminal type A: MCF-7, Luminal type B: BT474, HER-2 overexpression type: MDA-MB-453, Triple-negative type: MDA-MB-231) were used in order to investigate the effects of differential expression levels of Cosmc on cellular functions, with the protein level of Cosmc in these four cell lines measured by Western blot. As shown in Figure 1, the protein level of Cosmc significantly decreased in all of four BC cell lines in comparison with normal HMEC HBL-100 cell line (*P*<0.05). The protein level of Cosmc in the four BC cell lines ranked from the highest to the lowest was MCF-7 > BT474 > MDA-MB-453 > MDA-MB-231. These results demonstrated a low expression of Cosmc in BC cells, and additionally, Cosmc level was relatively higher in MCF-7 and BT474 cells and lower in MDA-MB-453 and MDA-MB-231 cells.

The article "Overexpression of Cosmc suppresses cell migration and invasion in different subtypes of breast cancer cells via Tn and T glycans" was retracted in 2022. Reasons: contaminated cell lines or tissues; duplicated images; signs of a paper mill; unreliable results or conclusions.

**Figure 1:** Cosmc is down-regulated in BC cell lines with different molecular types (**A**) The gray value of Cosmc protein band compared with the internal reference GAPDH band in normal HMEC HBL-100 cell line and BC cell lines, as measured by Western blot. (**B**) The protein level of Cosmc in normal HMEC HBL-100 cell line and BC cell lines; *P<0.05 vs*.* the HBL-100 cell line. Data were measurement data and expressed by mean ± standard deviation, and data comparison was analyzed by one-way analysis of variance with Tukey’s post hoc test. The experiments were repeated three times.

### Overexpression of Cosmc inhibits accumulation of Tn antigen by promoting T antigen expression

According to the findings mentioned above, the MCF-7 and BT474 cell lines, with relatively higher protein levels of Cosmc, were infected with sh-Cosmc lentiviral vector or sh-Cosmc NC. On the contrary, MDA-MB-453 and MDA-MB-231 with relatively lower protein level of Cosmc were both infected with oe-Cosmc lentiviral vector or oe-Cosmc NC. According to Western blot analysis and flow cytometry, MCF-7 (Figure 2A,B) and BT474 (Figure 2C,D) cells in the sh-Cosmc group showed lower protein levels of Cosmc and T antigen yet, displayed an increase in Tn antigen content compared with the sh-NC group (all *P*<0.05). The MDA-MB-453 (Figure 2E,F) and MDA-MB-231 (Figure 2G,H) cells from the oe-Cosmc group, displayed enhanced protein levels of Cosmc and T antigen, and a lower Tn antigen protein level (all *P*<0.05). These results provided evidence that overexpression of Cosmc could potentially inhibit accumulation of Tn antigen by increasing the levels of T antigen protein; this effect could be reversed by Cosmc knockdown.

**Figure 2:** Overexpression of Cosmc promotes T antigen protein levels via inhibition of Tn antigen expression (**A** and **B**) The relative protein of Cosmc (Western blot analysis), T antigen and Tn antigen (flow cytometry) to the internal reference GAPDH in MCF-7 cells after lentiviral vector transduction. (**C** and **D**) The relative protein of Cosmc (Western blot analysis), T antigen and Tn antigen (flow cytometry) compared with the internal reference GAPDH in BT474 cells after lentiviral vector transduction. (**E** and **F**) The relative protein of Cosmc (Western blot analysis), T antigen and Tn antigen (flow cytometry) compared with the internal reference GAPDH in MDA-MB-453 cells after lentiviral vector transduction. (**G** and **H**) The relative protein of Cosmc (Western blot analysis), T antigen and Tn antigen (flow cytometry) to the internal reference GAPDH in MDA-MB-231 cells after lentiviral vector transduction; *P<0.05 vs*.* the sh-NC group or the oe-NC group. Data were measurement data and displayed by mean ± standard deviation, and data comparison between two groups was evaluated by non-paired *t*-test. The experiments were repeated three times.

The article "Overexpression of Cosmc suppresses cell migration and invasion in different subtypes of breast cancer cells via Tn and T glycans" was retracted in 2022. Reasons: contaminated cell lines or tissues; duplicated images; signs of a paper mill; unreliable results or conclusions.

### Overexpression of Cosmc inhibits BC cell proliferation, migration, and invasion, while promoting cell apoptosis via regulation of Tn and T glycans

The cell proliferation, migration, invasion, and apoptosis of BC cell lines after different lentiviral vector transfection were assessed, and we then intended to study the effects of Cosmc overexpression or knockdown on the cellular functions of BC cells. The protein levels of proliferation markers Ki67 and PCNA and, of the proapoptotic proteins Bax and Bad in BC cell lines were determined by Western blot. The results (Figure 3A,B) showed that the levels of Ki67 and PCNA increased, while those of Bax and Bad decreased in MCF-7 and BT474 cells with the transfection of sh-Cosmc, in contrast with the sh-NC group (*P*<0.05). However, an opposite trend was noticed in MDA-MB-453 and MDA-MB-231 cells in the oe-Cosmc group in contrast with the oe-NC group (*P*<0.05).

**Figure 3:** Overexpression of Cosmc could inhibit proliferation, migration and invasion of BC cells while promoting cell apoptosis (**A** and **B**) The relative protein levels of Ki67, PCNA, Bax, and Bad to the internal reference GAPDH in BC cell lines as determined by Western blot. (**C** and **D**) The cell proliferation of BC cell lines followed lentiviral vector infection as evaluated by EdU staining (×200). (**E** and **F**) The cell migration of BC cell lines following lentiviral vector infection as assessed by a scratch test (×100). (**G** and **H**) The cell invasion of BC cell lines following lentiviral vector infection as determined by Transwell assay (×200). (**I** and **J**) The cell apoptosis of BC cell lines following lentiviral vector infection as examined by flow cytometry; *P<0.05 vs*.* the sh-NC group or the oe-NC group. Data were measurement data and displayed as mean ± standard deviation; data comparison between two groups was evaluated by non-paired *t*-test. The experiments were repeated three times.

As illustrated by EdU staining (Figure 3C,D), the MCF-7 and BT474 cells of the sh-Cosmc group exhibited higher numbers of EdU positive cells than the sh-NC group (*P*<0.05), while it was reciprocal in MDA-MB-453 and MDA-MB-231 cells of the oe-Cosmc group when compared with the oe-NC group (*P*<0.05).

Next, as demonstrated by the scratch test (Figure 3E,F), the migration ability of MCF-7 and BT474 cells was enhanced and the migration distance was increased in the sh-Cosmc group compared with the sh-NC group (*P*<0.05). In contrast, MDA-MB-453 and MDA-MB-231 cells displayed reduced migration ability as the migration distance was decreased in the oe-Cosmc group compared with the oe-NC group (*P*<0.05).

The article "Overexpression of Cosmc suppresses cell migration and invasion in different subtypes of breast cancer cells via Tn and T glycans" was retracted in 2022. Reasons: contaminated cell lines or tissues; duplicated images; signs of a paper mill; unreliable results or conclusions.

Next, as shown in the Transwell assay (Figure 3G,H), the invasion ability of MCF-7 and BT474 cells was improved as the number of invasive cells increased in the sh-Cosmc group in contrast to the sh-NC group (*P*<0.05). At the same time, the invasion ability of MDA-MB-453 and MDA-MB-231 cells was repressed and the number of invasive cells was decreased in the oe-Cosmc group compared with the oe-NC group (*P*<0.05).

Finally, flow cytometry (Figure 3I,J) demonstrated that the apoptosis rate of MCF-7 and BT474 cells was notably decreased in the sh-Cosmc group compared with the sh-NC group (*P*<0.05). At the same time, MDA-MB-453 and MDA-MB-231 cells displayed increased apoptosis rate in the oe-Cosmc group, compared with the oe-NC group (*P*<0.05). Collectively, these results suggested that overexpression of Cosmc could inhibit proliferation, migration and invasion of BC cells while promoting cell apoptosis, which could be reversed by silencing Cosmc.

### Overexpression of Cosmc inhibits tumorigenicity of BC cells *in vivo*

The MCF-7 and BT474 cell lines infected with sh-Cosmc lentiviral vector or sh-Cosmc NC, and MDA-MB-453 and MDA-MB-231 with oe-Cosmc lentiviral vector or oe-Cosmc NC were injected into nude mice with the purposes of investigating the effects of Cosmc on BC *in vivo*. At the end of experimentation of tumor xenografts in nude mice, the tumors were collected. The results showed that tumors removed from mice inoculated with MCF-7 and BT474 cells in the sh-Cosmc group displayed an increase in tumor volume (Figure 4A,B) and mass (Figure 4C), compared with the sh-NC group (all *P*<0.05). An opposite result was revealed in tumors removed from mice inoculated with MDA-MB-453 and MDA-MB-231 cells in the oe-Cosmc group compared with the oe-NC group (all *P*<0.05). These results demonstrated that Cosmc could suppress tumorigenicity of BC cells *in vivo*.

**Figure 4:** Overexpression of Cosmc inhibits BC cell proliferation and tumorigenicity while promoting apoptosis *in vivo* (**A**) Maps of tumors removed from mice; (**B**) tumor growth curve; (**C**) histogram of tumor mass; (**D** and **E**) the protein levels of Ki67, PCNA, Bax and Bad in tumor tissues as determined by Western blot analysis; (**F** and **G**) the proliferation of tumor cells as measured by EdU staining (×200); (**H** and **I**) the apoptosis of tumor cells as evaluated by flow cytometry; *P<0.05 vs. the sh-NC group or the oe-NC group; *N*=6. Data were measurement data and displayed as mean ± standard deviation. Data comparison between two groups was evaluated by non-paired *t*-test, and data comparison at different time points was analyzed by repeated measures analysis of variance with Bonferroni post hoc test.

The article "Overexpression of Cosmc suppresses cell migration and invasion in different subtypes of breast cancer cells via Tn and T glycans" was retracted in 2022. Reasons: contaminated cell lines or tissues; duplicated images; signs of a paper mill; unreliable results or conclusions.

Followingly, the protein levels of Ki67, PCNA, Bax, and Bad in tumor tissues were determined by Western blot. The results (Figure 4D,E) showed that the levels of Ki67 and PCNA increased, while Bax and Bad decreased in tumor tissues removed from mice inoculated with MCF-7 and BT474 cells in the sh-Cosmc group compared with the sh-NC group (*P*<0.05). Nevertheless, the tendency of the four aforementioned protein levels was reversed in tumor tissues of mice inoculated with MDA-MB-453 and MDA-MB-231 cells in the oe-Cosmc group in contrast to the oe-NC group (*P*<0.05).

Furthermore, the results of EdU staining (Figure 4F,G) and flow cytometry (Figure 4H,I) demonstrated that the number of EdU positive cells distinctively increased while the cell apoptosis rate decreased in the sh-Cosmc group when compared with the sh-NC group. As expected, this trend was reversed in the oe-Cosmc group in contrast with the oe-NC group (all *P*<0.05). All together, the above-mentioned results suggested that overexpression of Cosmc could inhibit BC cell proliferation while promoting apoptosis *in vivo*, which could be reversed by silencing Cosmc. The results were consistent with *in vitro* cell experiments.

## Discussion

BC remains a major cause of morbidity and mortality among the female population due to the high risk of regional and/or distal metastasis of the primary breast tumors [12]. Expression of normal O-glycans is critical for post-translational protein processing, and thus this process is closely associated with human health and homeostasis. Indeed, O-glycan truncation is related to cancer and other pathologies such as lack of Tn antigen, which is connected with a deficiency of active T antigen or Cosmc [13]. Our study explored the effects of Cosmc on the growth and metastasis of BC cells with different molecular types via regulation of Tn and T glycans. Furthermore, overexpression of Cosmc inhibited the generation of Tn antigen through enhancement of T antigen, which in turn led to the suppression of cell proliferation, invasion and migration of BC cells, along with increased apoptosis.

Initially, the data obtained in the present study revealed a low Cosmc expression in BC cell lines. One of the key mechanisms that can cause loss of Cosmc mRNA expression is hypermethylation of the Cosmc promoter region, which has been demonstrated in IgA nephropathy lymphocytes [14]. Interestingly, it has been suggested that epigenetic silencing of Cosmc may lead to abnormal expression of Tn antigen in human diseases, as shown in IgA nephropathy and many cancers [15,16]. In addition, a study by Warrier et al*.* has suggested that nanocarriers can be applied in anti-cancer therapies on the basis of the mechanism of antigen cross-presentation [17]. Cosmc deficiencies reduce T antigen activity by affecting T-synthase folding and, consequently, trigger the accumulation of Tn antigen in human tumors [18]. For example, Cosmc knockdown has been previously reported to enhance oncogenic properties in pancreatic cancer through an accumulation of aberrant O-glycosylation substrates and, increased Tn antigen expression was detected in Cosmc deficient pancreatic ductal adenocarcinoma (PDAC) cells [9]. In the human colorectal carcinoma cell line HT-29, abnormally expressed Cosmc could lead to Tn antigen expression [19]. Therefore, dysregulation of Cosmc is usually observed in many diseases as it plays as an anti-oncogene in multiple cancers and should be considered as drug target for BC.

The article "Overexpression of Cosmc suppresses cell migration and invasion in different subtypes of breast cancer cells via Tn and T glycans" was retracted in 2022. Reasons: contaminated cell lines or tissues; duplicated images; signs of a paper mill; unreliable results or conclusions.

Moreover, overexpression of Cosmc resulted in the rapid consumption of Tn antigen through an enhancement of T antigen expression. Tn antigen has been shown to have a close connection to tumor growth, differentiation, and metastasis, and thus, the levels of Tn antigen displayed in a tumor could be a crucial prognostic indicator [20]. Previous evidence has indicated that colorectal cancer cell lines expressing Tn presented with loss-of-function mutations in Cosmc or, reversible Tn antigen expression [21]. Cancer-specific mutations of the Cosmc gene could reduce the activity of T antigen and thus prevent synthesis of O-glycan core 1, which finally results in overexpression of the Tn antigen, thereby creating a cancer-specific epitope on the cell surface [22]. Tn antigen is almost undetectable in normal cells; however, mutation of the Cosmc gene could increase Tn antigen expression within certain cancers as a result of T-antigen inactivation, thus it is regarded as one of the most universal carbohydrate antigens that related to tumor [19]. Additionally, overexpression of Tn antigen has been found in BC and its expression is associated with the increased migratory potential of the MDA-MB-231 BC cell line [23]. It has also been reported that the levels of Tn antigen are negatively regulated by Cosmc and, furthermore, an elevation of Tn levels in cancer along with inflammation may be modulated via the cytokine–Cosmc signaling axis [24]. Thus, the regulation of Cosmc in balance of Tn–T antigen is associated with multiple cancers.

The article "Overexpression of Cosmc suppresses cell migration and invasion in different subtypes of breast cancer cells via Tn and T glycans" was retracted in 2022. Reasons: contaminated cell lines or tissues; duplicated images; signs of a paper mill; unreliable results or conclusions.

Finally, our results also found that the overexpression of Cosmc suppressed the expression of Ki67 and PCNA, while promoting that of Bax and Bad. Ki67 is a cell proliferation biomarker [25], and a high level of Ki67 in BC is related to ER negativity, HER2 positivity, higher grade and axillary lymph node involvement [26]. PCNA, with involvement in DNA excision repair and cell cycle control, exerts its major function in DNA replication, and an increased level of PCNA is linked to a shorter disease-free period and overall survival time in patients with BC [27]. Considering cell apoptosis, MCF-7 and BT549 human BC cells, which treated with Balsamin (a 28 kDa Type I ribosome-inactivating protein) to induce apoptosis, displayed increased levels of Bax, Bid, and Bad, which is related with Cosmc [28]. Similar to our research, an aforementioned study has indicated that cells with Cosmc knockdown exhibit increased proliferation and migration as well as decreased apoptosis, suggesting that the concomitant increase in Tn expression could play a significant role in various aspects of PDAC-derived cell metastatic and anti-apoptotic behaviors [9]. Overexpression of Cosmc results in suppression of Ki67 and PCNA and promotion of Bax and Bad, which then leads to the inhibition of proliferation, invasion and migration, and promotion of the apoptosis of BC cells.

Taken together, the key findings of the present study demonstrated that overexpression of Cosmc inhibited Tn antigen accumulation via T antigen promotion, thereby suppressing proliferation, invasion and migration of BC cells, along with higher rates of apoptosis. The present findings uncover a role of Cosmc as well as the molecular mechanisms underlying Cosmc function in tumor growth and metastasis in BC. Based on these findings, therapeutically targeting Cosmc may be a potential strategy to reduce BC occurrence or recurrence. However, whether this therapeutic target may be applicable in humans requires to be further verified by extensive clinical studies. Additionally, the findings provided in the present study are preliminary, indicating more studies in this area are required in the future.

## Data Availability

The datasets generated/analyzed during the current study are available.

## Abbreviations

BC: breast cancer
EdU: 5-ethynyl-2′-deoxyuridine
PDAC: pancreatic ductal adenocarcinoma
SPF: specific pathogen-free
sTn: sialyl-Tn
Tn: Thomsen nouvelle
TF: Thomsen-Friedenreich
